This article has been retracted.

# Psychological Shaping Function of Music Education to Cultivate the Subjective Initiative of University Students' Physical Training

**DOI:** 10.1155/2022/1832773

**Published:** 2022-09-10

**Authors:** Lin Zhou, Feng Yu

**Affiliations:** ^1^Department of Musicology, School of Music, Nanjing Normal University, Nanjing 210000, Jiangsu, China; ^2^Department of Musicology, School of Music, Jiangsu Normal University, Xuzhou 221116, Jiangsu, China

## Abstract

The purpose of university students' physical training (PT) is to make university students have a good exercise habit and improve their willpower while enhancing their immunity. However, because many university students are not active in physical exercise, who worry about sweating during exercise, with low requirements for physical exercise, the subjective motivation of university students in PT is poor. Music education (MUE) is a new educational model. Through the correct guidance of university students' psychology, the inner health of university students can be enhanced, so that university students can carry out PT with a positive attitude. MUE is applied to university students' PT to cultivate the subjective initiative of university students' PT by shaping the psychology of university students. This paper evaluates the influence of the psychological shaping of MUE on the subjective initiative of university students' PT through the analytic hierarchy process (AHP). The experimental results showed that the top three weights of the evaluation indicators were the effect of MUE, the effect of university students' music learning, and the psychological state of university students. Comparing and analyzing the three indicators of MUE and traditional education, the average values of the two education methods in the subjective initiative of university students' PT were 61.3% and 34.2%. Compared with traditional education, MUE can effectively improve the effect of PT. Therefore, MUE can improve the subjective initiative of university students' PT through the psychological guidance of university students, so that university students can exercise actively, improving the effect of PT.

## 1. Introduction

University physical exercise is to cultivate university students to have a strong body and cultivate the habit of lifelong exercise for university students. However, due to the lack of attention of universities to students' PT and the inactiveness of university students to PT, university students' physical fitness is low. The decline in the physical quality of university students leads to problems such as inattention and low learning efficiency in class. The main factor that causes university students not to be active in PT is the decrease of the subjective initiative of university students to PT. PT subjective initiative means that university students can have a positive and active influence on PT after receiving the feedback of PT. The way to enhance the subjective initiative of university students' PT is to improve the university students' in-depth understanding of PT and to enhance the psychological emotions of university students' PT. MUE can not only guide the mentality of university students in physical exercise but also change the attitude of university students to physical exercise; thus, improving the subjective initiative of university students in PT. Exploring the influence of the psychological shaping function of MUE on the subjective initiative of university students' PT can effectively improve the enthusiasm of university students for PT and improve the efficiency of college sports training.

The physical quality of university students is getting worse and worse. Some researchers have studied the subjective initiative of university students' PT to improve the physical quality of university students. Among them, Jung's and Yeun research pointed out that by cultivating the individual's subjective initiative university students' PT, the interest of university students in PT can be improved [1]. Kim and Lee said that the subjectivity of university students' PT can stimulate the potential of students' PT and increase the effectiveness of university students' PT [2]. Lee and Jang divided university students into two groups, among which students with high subjective motivation in university sports training have stronger physique [3]. Zhang's research showed that improving the subjective motivation of university students' PT can enhance the physical fitness of university students [4]. Liang indicated that the subjective initiative of university students' PT is the main factor affecting the effect of university students' PT. Higher subjective motivation can improve the effect of physical training [5]. Although improving the subjective activity of university students' PT improves the training effect and enhances the physique of university students, there is a scarcity of study on university students' psychology.

MUE has the function of psychological shaping. Using MUE can cultivate the individual's subjective initiative university students' PT. Among them, Wicaksono said that long-term MUE can make the psychology of university students healthier and help cultivate the subjective initiative of university students in PT [6]. Payne et al. concluded that MUE can make the mental state of university students healthier by surveying the mental health of MUE. Music education can improve the subjective initiative of college students' physical training [7]. Zhang and Liu's application of MUE to university students enhanced the enthusiasm of university students for sports training [8]. Lee's research showed that MUE can shape the psychology of university students and has a positive effect on university students' PT [9]. Orlova, through his research on university students' music psychology, said that scientific MUE can effectively improve the subjective initiative of university students' PT [10]. Although MUE can improve the enthusiasm of university students' PT through the psychological construction of university students, there is a lack of specific evaluation models to quantitatively analyze the subjective initiative of MUE and university students' PT.

MUE has the function of shaping psychology. The MUE is applied to the education of university students, and the relationship between MUE and the subjective initiative of university students' PT is analyzed through the AHP, so as to improve the subjective initiative of university students' PT. The innovations of this paper are reflected in the following aspect: using the AHP to quantitatively analyze the subjective initiative of MUE and university students' PT, the factors that can improve the subjective initiative of university students' PT are obtained.

## 2. AHP Evaluation

Music is a discipline and the embodiment of human artistic wisdom, which is gradually applied from an artistic act to the field of education. MUE can adjust the psychological state of university students through soothing music [11]. MUE can psychologically affect the subjective initiative of university students' PT, enhance the physique of university students, and promote the all-round development of university students [12].  Figure 1 shows the structure of the psychological impact of MUE on the subjective initiative of university students' PT.

In Figure 1, music affects the psychology of university students in the form of education. It actively guides the psychology of university students, enhancing the subjective initiative of university students in PT, thereby making college students more active and effective in participating in various sports.

### 2.1. Subjective Initiative

Subjective initiative refers to people in the environment, through their own subjective consciousness, make corresponding responses to the external environment [13]. In the sports training mode, university students are in a passive position to receive knowledge. When university students do not actively carry out sports training, the training will become meaningless. In sports training, no one supervises students, and university students have low requirements on themselves. There are also some university students who are reluctant to do PT because they are afraid of getting dirty and sweating. These negative attitudes towards PT make university students inefficient in PT.

The improvement of the subjective initiative of university students in PT can make university students be more active in PT, which also can promote their body and mental health, exercise their willpower, and enhance their physical quality. There are three main ways to cultivate the subjective initiative of university students' PT.

#### 2.1.1. Implementing Music Teaching

Music teaching relieves the psychology of university students through beautiful music, relieves pressure on university students on a psychological level, and makes university students relax wholeheartedly, which can improve the subjective initiative of university students' PT.

#### 2.1.2. Improving University Students' Awareness of PT

Many university students have a very narrow cognition of PT, just to cope with the school's physical examination [14]. When teaching PT to university students, physical education teachers can explain some more physical knowledge.

#### 2.1.3. Carrying Out More Sports Training Activities in Universities

Large-scale sports training activities can make university students participate in sports training, so that university students in sports activities feel a feeling of responsibility and mission. The subjective initiative of college students' physical training is also improved.

### 2.2. AHP

The influence of the psychological shaping function of MUE on the subjective initiative of university students' PT is a multifactor problem. The analysis of subjective initiative in traditional MUE can only be an artificial judgment mode. The way of judgment is usually carried out in the form of a questionnaire, but the results of artificial judgment are inaccurate, which cannot quantitatively analyze the influencing factors [15].

AHP is a quantitative analysis method and makes it scientific and reasonable to evaluate the subjective initiative of university students' PT through the weight analysis of each factor [16]. AHP mainly decomposes the goals to be achieved into various factors. Then it performs hierarchical processing on the decomposed factors and calculates the weight analysis of each factor to achieve the goal by comparing in turn. The structure of AHP is shown in Figure 2.

The target layer is the goal to be achieved by the system, which is represented by the subjective initiative *X* of university students' PT in this paper. The target layer can be divided into the criterion layer Y, and the criterion layer can be further divided into the index layer Z. The final specific evaluation is to evaluate the influence of each index on the subjective initiative of university students' PT [17].

In the AHP, the weight of each factor affecting the experimental target is analyzed mainly by constructing a judgment matrix. When constructing the judgment matrix, it is necessary to quantitatively estimate and score the factors. The scoring is done by the subjective initiative judges of professional university sports training. Ratings are based on numbers 1-9. A larger value represents a greater correlation, while the inverse of the number indicates a small correlation [18]. The scoring table of the matrix is shown in Table 1.

The formula of the judgment matrix is expressed as

(1) $$\begin{array}{c} B={\left(b_{ij}\right)}_{n\times n}. \end{array}$$

In formula 1, *b*_ij_ is the score at row *i* and column *j* of the matrix.

The judgment matrix of the AHP is the comparative relationship between the factors, and the relative weight of each factor can be obtained through the analysis of the judgment matrix.

The relative weight calculation of each factor can be calculated by the arithmetic average method, and the average of each column vector in the judgment matrix represents the weight of the corresponding factor. The calculation process of the arithmetic average method is as

(2) $$\begin{array}{c} b_{i}=\frac{b_{i1}+b_{i2}+\cdots +b_{in}}{n}. \end{array}$$

In formula 2, *b*_i_ represents the *i*-th column vector of the judgment matrix.

The calculated factor weights also need to be effectively tested. The effective test is to make the calculated weights credible and avoid discrepancies between the calculated factor weights and the facts. The index formula for the valid test is as

(3) $$\begin{array}{c} I=\frac{\mu_{\max}-n}{n-1}. \end{array}$$

In formula 3, *μ*_max_ is the largest eigenvalue of the corresponding matrix.

The formula for determining the percentage of valid tests is as

(4) $$\begin{array}{c} R=\frac{I}{RI}. \end{array}$$

In formula 4, *RI* represents the effective test index of the matrix.

When *R* < 0.1, it means that the matrix of judgment is correct, and the weight can be used as the judgment basis for the experiment. On the contrary, the judgment matrix is invalid.

## 3. PT Experiment Design and Data

### 3.1. Experimental Data

In order to analyze the indicators of subjective motivation in MUE and university students' PT, the experiment requires a questionnaire survey of professionals. 150 professionals were surveyed for MUE and university sports training. Among them, there were 50 music teachers, 50 psychology experts, and 50 university physical education teachers. They investigated the indicators that they believed that MUE could affect the subjective of university students' PT [19]. The survey results are shown in Table 2.

In Table 2, the evaluation indicators agreed by the investigators with the highest proportion were the effect of music teaching and the attitude of university students to PT. The lowest proportion was MUE goals and MUE methods accounting for 92.0%. Each index in Table 2 had an approval rate of more than 92%. The evaluation indicators shown in Table 2 have evaluation significance and can be used as indicators to evaluate the influence of MUE on the subjective initiative of university students' PT [20].

### 3.2. Experimental Design

This paper uses AHP to study the relationship between MUE and the subjective initiative of university students' PT. Through the judgment matrix, it analyzes which factors can significantly enhance the subjective initiative of university students' PT and then analyzes the changes that the improvement of university students' PT subjective initiative can bring to university students' PT [21].

A judgment matrix is constructed for each index in Table 2. It includes the judgment matrix of target *X* for criterion layer *Y*, criterion layer *Y* for index layer. It is supposed that MUE is *Y*_1_, and mental shaping is *Y*_2_.

Then, the judgment matrix of target *X* for criterion layer *Y* is shown in Table 3.

*μ*_max_=2 can be obtained by solving the maximum eigenvalue of the matrix in Table 3. In a second-order matrix, *RI*=0, so the matrix passes the validity test.

The judgment matrix of MUE *Y*_1_ to indicator *Z* is shown in Table 4.

*μ*_max_=6.5 can be obtained by solving the maximum eigenvalue of the matrix in Table 4.

Substituting it into formula 4, the following formula can be calculated:

(5) $$\begin{array}{c} R=\frac{0.1}{1.26}=0.079. \end{array}$$

In formula 5, *R* < 0.1, so the matrix passes the validity test.

The judgment matrix of MUE *Y*_2_ for indicator *Z* is shown in Table 5.

Similarly, *R*=0.0418 < 0.1 can be obtained through the validity test of Table 5, so the matrix passes the validity test.

## 4. Results

### 4.1. Weight of Each Factor

The weight of each evaluation factor represents the influence of each factor on the subjective initiative of PT. The weight of each factor is calculated by calculating each column vector in the judgment matrix, and the calculation process applies formula 2 in this paper. The weight calculation results of each factor are shown in Figure 3.

In Figure 3, factors 1-9 represent the evaluation indicators from the top to bottom in Table 2, respectively. The weight of each factor was not very different, indicating that each evaluation index in Table 2 had a significant influence on the subjective initiative of university students' PT [22]. Among them, the weight of MUE effect was the largest, 0.135, followed by the weight of university students' music learning effect of 0.124, and the third was the weight of university students' psychological state of 0.115.

### 4.2. Effect of MUE

The effect of MUE can have the greatest influence on the subjective initiative of university students' PT. By setting the gradually increasing MUE effect, the impact of MUE effect on the subjective initiative of university students' PT and the effect of university students' PT can be judged [23]. The effect of MUE effect is shown in Figure 4.

In Figure 4, the gradual improvement of the teaching effect showed that the music teaching mode had a positive influence on the subjective initiative of university students' PT. Under the best conditions of MUE, the subjective initiative of university students' PT reached 86%, while traditional teaching at the same time only reached 55%. The average PT effect of university students under MUE and traditional education was 57.6% and 32.0%, respectively. Improving the effect of MUE can significantly improve the subjective motivation and effect of PT of university students [24].

### 4.3. Influence of Effect of University Students' Music Learning

The music learning effect of university students represents the learning ability of university students in music teaching. By setting different music learning effect gradients for different students, the impact of university students' music learning effect on the subjective initiative of university students' PT can be judged. The influence of university students' music learning efficiency is shown in Figure 5.

In Figure 5, when the music learning effect was less than 40%, the subjective initiative and PT effect of university students' PT produced by the two education models were not much different [25]. However, the increase in the effect of music learning makes the growth trend of university students' PT subjective initiative and PT effect more and more large. The average subjective motivation was 47.6%, and the average PT effect was 66.4%. But, the subjective initiative and effect of PT of university students under traditional education were very poor. The averages were 32.6% and 50.0%.

### 4.4. Influence of University Students' Psychological State

MUE can guide the psychological state of university students. The condition of mind of university students can effectively affect the subjective of university students' PT. The psychological states of university students with different gradients were set, which were set as 5 grades: extremely poor, poor, medium, good, and excellent. The condition of mind of university students affected the results of the subjective initiative of university students' PT and PT effects, as shown in Figure 6.

In Figure 6, in both education modes, the gradient growth of mental state increased the subjective motivation and effect of PT of university students. However, the average effects of the two educational models were quite different [26,27]. The subjective motivation of university students' PT and the average subjective motivation of the two education models was 76.6% and 40%, respectively. The effect of university students' PT and the average PT effects of the two education models were 78.6% and 40.2%, respectively.

Music education is a new type of education, which can actively guide students through psychological analysis. Applying music education to college students' physical training analyzes the influence weight of music education on college students' physical training by AHP and determines how music education can cultivate the subjective initiative of college students' physical training according to the analyzed influencing factors. Therefore, it can improve the subjective initiative of college students' physical training and improve the effect of college students' physical training.

## 5. Conclusions

This article investigates the impact of the psychological shaping function of MUE on the subjective initiative of university students' PT. Through qualitative analysis of relevant experts and quantitative analysis of relevant indicators using AHP, this paper analyzes its influence on the subjective initiative of university students' PT. The maximum weight of MUE effect was 0.135. The second weight was the music learning effect of university students. The third weight was the condition of mind of university students. The first three indicators of weight were set as gradients, and it was found that MUE can enhance the subjective initiative of university students' PT and the effect of PT by improving the effect of MUE, the learning effect of university students, and the psychological state of university students. MUE and traditional education were compared. The average subjective motivation of university students' PT under the two education modes was 61.3% and 34.2%, respectively. The effects of PT were 67.5% and 40.7%, respectively. This paper analyzes the influencing factors of music education on college students' subjective initiative by the method of analytic hierarchy. By analyzing the weight of the influencing factors, and analyzing the influencing factors of music education and traditional education, music education can improve the subjective initiative of college students' physical training. By shaping the psychology of university students, MUE can relax the body and mind of university students and improve the enthusiasm of university students' psychology. MUE can effectively improve the subjective of university students' PT and the efficiency of PT. However, the factors analyzed in this paper are not comprehensive enough to cover all the effects of MUE on the subjective initiative of university students' PT. Therefore, it will be the direction of future research to expand the analysis factors of MUE on the subjective initiative of university students' PT.

## Figures and Tables

**Figure 1:** MUE psychologically affects the subjective initiative of university students' PT.

**Figure 2:** AHP structure diagram.

**Figure 3:** Weight diagram of each factor.

**Figure 4:** Results of the effect of MUE. (a) Subjective initiative. (b) Effect of PT.

**Figure 5:** Results of music learning effects. (a) Subjective initiative. (b) Effect of PT.

**Figure 6:** Influence of university students' psychological state. (a) Subjective initiative. (b) Effect of PT.

**Table 1:** Scoring table for the matrix.

Score	Significance (importance of a factor)	Grade
1	*f* 1 = *f* 2	Level 0
2	*f* 1 > *f* 2	Level 1
3	*f* 1 > *f* 2	Level 2
4	*f* 1 > *f* 2	Level 3
5	*f* 1 > *f* 2	Level 4
6	*f* 1 > *f* 2	Level 5
7	*f* 1 > *f* 2	Level 6
8	*f* 1 > *f* 2	Level 7
9	*f* 1 > *f* 2	Level 8
1/9	*f* 1 < *f* 2	Level −8
1/8	*f* 1 < *f* 2	Level −7
1/7	*f* 1 < *f* 2	Level −6
1/6	*f*1 < *f* 2	Level −5
1/5	*f* 1 < *f* 2	Level −4
1/4	*f* 1 < *f* 2	Level −3
1/3	*f* 1 < *f* 2	Level −2
1/2	*f* 1 < *f* 2	Level −1

**Table 2:** Evaluation index questionnaire results.

Level	Index	Number of people (person)	Proportion (%)
Musical education	The effect of MUE	148	98.7
	MUE content	140	93.3
	MUE management	142	94.7
	MUE goals	138	92.0
	Methods of MUE	138	92.0
	Level of MUE	140	93.3
Psychological shaping	Mental state of university students	146	97.3
	University students' attitudes to PT	148	98.7
	The effect of university students' music learning	144	96.0

**Table 3:** Judgment matrix of target *X* for criterion layer *Y*.

*X*	*Y *_1_	*Y *_2_
*Y *_1_	1	2
*Y *_2_	1/2	1

**Table 4:** Judgment matrix of MUE *Y*_1_ for indicator *Z*.

*Y *_1_	*Z *_1_	*Z *_2_	*Z *_3_	*Z *_4_	*Z *_5_	*Z *_6_
*Z *_1_	1	1/6	1/3	1	1/3	2
*Z *_2_	6	1	3	4	3	4
*Z *_3_	3	1/3	1	2	1/4	4
*Z *_4_	1	1/4	1/2	1	1/3	1
*Z *_5_	3	1/3	4	3	1	3
*Z *_6_	1/2	1/4	1/4	1	1/3	1

**Table 5:** Judgment matrix of MUE *Y*_5_ for indicator *Z*.

Y_1_	*Z *_7_	*Z *_8_	*Z *_9_
*Z *_7_	1	3	1
*Z *_8_	1/3	1	1/2
*Z *_9_	1	2	1

## Data Availability

The data used to support the findings of this study are available from the corresponding author upon request.
